# Functional annotation of extensively and divergently expressed miRNAs in suprachiasmatic nucleus of *Clock*^Δ19^ mutant mice

**DOI:** 10.1042/BSR20180233

**Published:** 2018-12-07

**Authors:** Yanli Wang, Ke Lv, Hailong Chen, Mei Zhao, Guohua Ji, Yongliang Zhang, Hongqing Cao, Guanghan Kan, Yinghui Li, Lina Qu

**Affiliations:** 1 School of Life Sciences, Northwestern Polytechnical University, Xian, Shaanxi 710072, China; 2 State Key Laboratory of Space Medicine Fundamentals and Application, China Astronaut Research and Training Center, Beijing 100094, China; 3 Institute of Psychology, Chinese Academy of Sciences, Beijing 100101, China

**Keywords:** Circadian rhythms, Clock mutation, microRNA, Suprachiasmatic nuclei

## Abstract

Circadian locomotor output cycles kaput protein (CLOCK) is a core transcription factor of complex integrated feedback loops in mammalian circadian clock. More genes have been reported to be regulated by CLOCK, however little is known about the role of CLOCK-mediated miRNAs. To dissect this, we used microarray analysis to measure miRNAs expression in suprachiasmatic nuclei (SCN) of wild-type (WT) and *Clock^Δ19^* mutant mice at two different time points. We found that miRNAs regulation in two time points was extensive (nearly 75% of the miRNAs expressed at each time point), and very little overlap, with only six miRNAs in common. Besides this, the predicted CLOCK regulated miRNAs at two time points participated in extremely diverse pathways. We validated nine miRNAs (miR-125a-3p, miR-144, miR-199a-5p, miR-199b*, miR-200a, miR-200b, miR-203, miR-449a, and miR-96), which were involved in the same signaling pathway-hippo signaling pathway. The rhythms of these miRNAs showed a broad distribution of phase, amplitude, and waveform in *Clock* mutation. And further analysis indicated that there may be three models of miRNA-mediated circadian rhythms and hippo signaling pathway. MiRNA, the small player, may play a hub role in connecting circadian rhythms and other pathways via its multiple target genes networks.

## Introduction

In mammals, circadian rhythms are generated by a central pacemaker in the suprachiasmatic nuclei (SCN) of the hypothalamus [1]. The molecular mechanism of the circadian oscillator as a transcriptional–translational feedback loop, constructed by genes such as *clock, bmal1, per1-3, cry1-2*, and *nr1d1-2*, unraveled by genetic analysis in mammals [2–4]. The transcriptional activators, such as CLOCK (circadian locomotor output cycles kaput) and BMAL1 (brain muscle arnt-like1), regulate other core genes expression by interacting with enhancer elements termed as E boxes [5].

After the core transcriptional molecular mechanism was defined, post-transcriptional regulation was increasingly recognized as an important process in the molecular feedback loops of circadian rhythms. MiRNAs as a kind of small RNA amongst non-coding RNAs, mostly bind to the 3′-UTR of target mRNAs, where they function to block translation or decrease mRNA stability [6]. Cheng and colleagues [7] found that miR-219 and miR-132 displayed circadian expression pattern in the SCN and identified several potential mRNA targets. Furthermore, circadian period length and light-dependent clock resetting were altered in the absence of miR-219 and miR-132, respectively [8]. However, the identification of CLOCK controlled genes (CCGs), especially CLOCK-regulated miRNA, and their efficacy to target functional genes, largely need to be uncovered.

In the present study, to identify CLOCK-related miRNAs in central circadian oscillator, we performed microarray analysis in RNA sample isolated from SCN of wild-type (WT) and *Clock*^Δ19^ mutant mice at two zeitgeber time (ZT2 and ZT14), which the CLOCK transcriptional activity was maximal and minimal at ZT2 and ZT14, respectively. Then, the changed miRNAs in *Clock^Δ19^* mutant mice were integrated to DIANA-miRpath v.3 to analyze the signaling pathway. Moreover, nine miRNAs, which were related to hippo signaling pathway were verified. Consequently, we raised three models of miRNA-mediated circadian rhythms and hippo signaling pathway to facilitate further functional study of post-transcriptional regulation in circadian rhythms. And to test the hypothesis model, the expression level of PER2 was also analyzed by overexpressing or inhibiting miR-199a-5p, miR-449a, and miR-96.

## Materials and methods

### Ethics statement

In the present study, all procedures used in animals were conducted in compliance with animal protection protocol as approved by the Institutional Animal Care and Use Committee in China and all the experimental procedures were approved by the Committees of Animal Ethics and Experimental Safety of China Astronaut Research and Training Center.

### Animals, conditions, and bio-sample collections

The animals were 6–7-week-old *Clock^Δ19^* mutant mice and age- and sex-matched WT C57BL/6J control mice. *Clock* mutant mice (*Clock*^Δ19^) were acquired from Institute of Psychology, Chinese Academy of Sciences, Beijing, China. All animals were housed in a temperature (22–25°C) and humidity (55 ± 5%) controlled room with food and water freely available in the home cages. Before the bio-sample collection procedures, all mice were individually caged for 2 weeks and maintained under IVC conditions with 12-h:12-h light/dark cycle, lights on at 7:00 a.m. (referred to as ZT point 0, ZT0) and lights off at 7:00 p.m. (referred to as ZT12). At ZT2 and ZT14 on the last day of 2 weeks, the animals were killed with dry ice asphyxia method. The SCN were dissected, quickly frozen, and stored in liquid nitrogen.

### RNA labeling and microarray hybridization

According to the Illumina’s protocol of mirVana™ RNA Isolation Kit (Qiagen, Germany), the three RNA samples at each time point were mixed and extracted. Then the RNAs were amplified using the Ambion TotalPrep RNA Amplification kit with biotin-UTP (Enzo) labeling. RNA labeling and microarray hybridization were analyzed by Shanghai OE Biotech. Co., Ltd. The Fold Change Absolute (FCA) larger than or equal to 2 was considered to have evident difference. We used the HemI [9], an online tool to set up the heatmap of the changed miRNAs in SCN of *Clock* mutant mice.

### Signaling pathway analysis

For the analysis of miRNAs pathway, the altered miRNAs were integrated into DIANA-miRpath v.3 [10].

### Quantitative real-time reverse transcriptional PCR

The expression of common miRNAs was measured by quantitative real-time RT-PCR. Briefly, after extraction of the RNAs from SCN with the TRIzol regent (Invitrogen, U.S.A.), the cDNAs were produced using One Step PrimeScript® miRNA cDNA Synthesis Kit (Cat# D350A, TaKaRa). Next, the cDNAs were used as the templates for the qPCR, which was performed using the SYBR® Premix Ex Taq™II (Cat# DRR820A, TaKaRa). The sequences of primers used for qRT-PCR were as follows (Table 1). Amplification data were analyzed using the comparative threshold (2^−ΔΔ*C*^_C_) method after normalization to U6.

**Table 1:** The primers used for qRT-PCR analysis

Gene	Primer sequences (5′–3′)	Gene	Primer sequences (5′–3′)
*miR-125a-3p*-F	ACAGGTGAGGTTCTTGGGAGCC	*miR-203*-F	GTGAAATGTTTAGGACCACTAG
*miR-144*-F	TACAGTATAGATGATGTACT	*miR-449a*-F	TGGCAGTGTATTGTTAGCTGGT
*miR-199a-5p*-F	CCCAGTGTTCAGACTACCTGTTCA	*miR-96*-F	TTTGGCACTAGCACATTTTTGCT
miR-199b*-F	CCCAGTGTTTAGACTACCTGTTC	*U6*-F	CTCGCTTCGGCAGCACA
*miR-200a*-F	TAACACTGTCTGGTAACGATGT	*U6*-R	AACGCTTCACGAATTTGCGT
*miR-200b*-F	TAATACTGCCTGGTAATGATGA		

The reverse primer of miRNAs referred to the manual of One Step PrimeScript® miRNA cDNA Synthesis Kit (Cat# D350A, TaKaRa). Abbreviations: F, forward; R, reverse.

### miRNAs regulatory network

To evaluate the interactive relations of miRNAs, circadian rhythms, and hippo signaling pathway, circadian genes and the prediction target genes of miRNAs were mapped to an online tool, STRING (version 10.0) [11]. The protein–protein interaction (PPI) information were obtained from STRING, and then, the Cytoscape [12] was used to construct the network. Also, Molecular Complex Detection (MCODE), one plug-in unit of Cytoscape was set to screen the models of PPI network. The criteria were set as follows: MCODE scores >5 and number of nodes >10.

### Cell culture, miRNAs transfection, and Western blot

NIH-3T3 mouse fibroblast cells were maintained in high-glucose Dulbecco modified Eagle medium (Sigma, U.S.A.) containing 10% FBS (Gibco) under standard cell culture conditions of 37°C, 5% CO_2_, and 95% humidity. miR-199a-5p, miR-449a, miR-96 mimics, and non-targetting miRNA mimics (negative control), and antisense mimics, scrambled antisense miRNA negative control were transfected into NIH-3T3 cells with Lipofectamine 2000 according to the manufacturer’s instructions, separately. After 48 h of transfection, cells were lysed in RIPA buffer (Sigma, U.S.A.). Twenty micrograms of protein extract was loaded on 15% tris-polyacrylamide gels. The proteins were then transferred to nitrocellulose membrane (Milipore, U.S.A.) and incubated with mouse anti-PER2 (Abcam, U.S.A.) overnight at 4°C. After washing, the membrane was incubated for 1 h with secondary antibodies at room temperature, and treated with Western blotting luminol reagent (Santa Cruz Biotechnology, U.S.A.) for chemiluminescence detection of protein bands.

### Statistical analysis

All numerical data were expressed as the mean ± S.D. Statistical differences between two groups were determined by the Student’s *t* test. Difference with *P*<0.05 was considered statistically significant.

## Results

### Differentially expressed miRNAs were mostly distinct at two time points

To identify the putative CLOCK regulated-miRNAs in central pacemaker, we analyzed the miRNAs profile in SCN of *Clock*^Δ19^ mutant and WT mice at two different time points using microarray. Of 651 miRNAs, 39 differentially expressed miRNAs (22 miRNAs at ZT2 and 23 miRNAs at ZT14) were found in SCN of *Clock* mutant mice (Figure 1A). The miRNAs’ expression profiles in SCN at two ZTs had very little overlapping, with only six miRNAs in common (Figure 1B).

**Figure 1:** The expression profile of changed miRNAs in SCN of *Clock*^∆19^ mutant mice (**A**) The heatmap of changed miRNAs in SCN of *Clock* mutant mice at two ZTs (ZT2 and ZT14). (**B**) Shared in common and differentially expressed miRNAs between two different zeitgebers.

### Hippo signaling pathway was unraveled dominant amongst 15 mostly shared regulatory pathways

The divergence of the expression of miRNAs in SCN suggests a specialized role of miRNAs at each time, but the sheer extent of miRNAs regulation in both time points implies a broad function. To address this apparent contradiction, we first used the Tarbase to analyze the targets of single miRNA, and then used the DIANA TOOLS-miRpath v.3 to analyze the miRNAs pathway. The results showed that three miRNAs targetted circadian genes (miR-125a-3p targets PER3, miR-449a and miR-484 target PER2). Comparison of the overlap between two time points revealed 15 signaling pathways in common (Figure 2). Interestingly, most of differentially expressed miRNAs (14 miRNAs of all 22 at ZT2 and 15 miRNAs of all 23 at ZT14) were shown in hippo signaling pathway.

**Figure 2:** miRNA-regulated pathways in SCN of *Clock* mutant mice at ZT2 and ZT14 Red color represents miRNAs shared in common at ZT2 and ZT14. Blue color represents pathway shared in common at ZT2 and ZT14.(**A**) miRNAs-regulated pathways in SCN of Clock mutant mice at ZT2. (**B**) miRNAs-regulated pathways in SCN of Clock mutant mice at ZT14.

### *Clock* mutation changed the rhythms of miRNAs’ expression levels

To further investigate the putative CLOCK-regulated miRNAs, we consecutively collected the SCN from WT and *Clock^Δ19^* mutant mouse during 24 h at 4-h interval to determine the expression level of nine miRNAs in hippo signaling pathway (miR-125a-3p, miR-144, miR-199a-5p, miR-199b*, miR-200a, miR-200b, miR-203, miR-449a, and miR-96). The expression of miR-199a-5p, miR-200a, miR-200b, and miR-96 were up-regulated under *Clock* mutant conditions. The rhythm oscillations of these miRNAs showed a broad distribution of phase, amplitude, or waveform (Figure 3A–I). We further analyzed the fold change of microarray and qPCR results. As shown in Figure 3J, the qPCR fold change of these miRNAs was consistent with the above microarray results, except the miR-199b* at ZT2 and miR-449a at ZT14.

**Figure 3:** Temporal patterns of putative clock-regulated miRNAs in the mouse SCN In (**A**–**I**), *Clock*^∆19^ compared with WT, *n*=5 of each group with *P<0.05 and **P<0.01. In (**J**), the y-axis represents the relative fold change, value greater than zero represents the up-regulation and the value less than zero represents the down-regulation. The relative fold change (FC) of microarray was analyzed by the FC of *Clock* mutant and WT mouse with mathematical formula log2 ^FC(^*^Clock^*^)/FC(WT)^. The relative fold change of qRT-PCR was analyzed by the value after normalization to U6 with the comparative threshold method. If the value of Clock mutant more than WT mouse, the up-regulation fold change was calculated with the formula 2^−ΔΔ*C*^_C_^(^*^Clock^*^)^/2^−ΔΔ*C*^_C_^(WT)^. The down-regulation FC was considered when the value of Clock mutant less than WT mouse and analyzed by the mathematical formula 2^−ΔΔ*C*^_C_^(WT)^/2^−ΔΔ*C*^_C_^ (Clock)^.

### CLOCK may regulate miRNAs via E-box element

More studies implied that a large number of genes might be regulated directly by CLOCK via the E-box. Thus, it was interesting to explore the gene family and the possibility that if these miRNAs had canonical E-box element. We found that these miRNAs were mainly involved in four gene families. miR-200a, miR-200b, miR-200c, and miR-429 belong to miR-8 gene family. Let-7a*, let-7b*, let-7d*, and let-7f* were involved in let-7 gene family. MiR-669b, miR-669d, and miR-467c expanded into a family of miR-467 gene family. And miR-199 gene family included miR-199a-3p, miR-199a-5p and miR-199b*. By analyzing the 5′ flank sequence of these miRNAs, we found a canonical E-box (CACGTG) in 12 miRNAs (Table 2).

**Table 2:** The chromosome position, gene family, and E-box position in 5-kb genome sequences upstream of miRNAs

miRNA	Chromosome	Gene family	E-box (kb)	miRNA	Chromosome	Gene family	E-box (kb)
mmu-miR-200a	4	miR-8	2.932	mmu-miR-144	11	miR-144	3.262
mmu-miR-200b	4	miR-8	3.706	mmu-miR-145	18	miR-145	2.315
mmu-miR-200c	6	miR-8	2.048	mmu-miR-199b*	2	miR-199	0.948
mmu-miR-429	4	miR-8	1.937	mmu-miR-203	12	miR-203	3.502
mmu-let-7a*	13	Let-7	1.950	mmu-miR-375	1	miR-375	3.760
mmu-let-7f*	13	Let-7	1.595	mmu-miR-449a	13	miR-449	1.244

### *Clock* and hippo signaling pathway

To get a more comprehensive understanding of the roles of the changed miRNAs between circadian rhythms and hippo signaling pathway, we used the core circadian genes (such as *clock, bmal1, per1, per2, per3, cry1, cry2, nr1d1*, and *nr1d2*), nine miRNAs (miR-125a-3p, miR-144, miR-199a-5p, miR-199b*, miR-200a, miR-200b, miR-203, miR-449a, and miR-96) and their putative target genes in hippo signaling pathway to construct the miRNAs regulatory network. As shown in Figure 4, two miRNAs targetted circadian genes (miR-449a targetted Per2 and miR-125a-3p targetted Per3). The *csnk1e* gene, which was regulated by miR-125a-3p, possessed a very important interaction with circadian rhythms and hippo signaling pathway. In addition, four genes were regulated by two miRNAs (both miR-200a and miR-200b regulate Tgfβ1, both miR-449a and miR-125a-3p target Ccnd1, both miR-125a-3p and miR-203 regulate Tcf7l2 or Ppp2ca).

**Figure 4:** Circadian rhythms and hippo signaling pathway Pink color represents the core circadian genes, red color represents the miRNAs and blue color represents the miRNAs targeting genes related to hippo signaling pathway. Triangles represent the core gene to connect circadian rhythms and hippo signaling pathway. Parallelogram and V represent the core two models in hippo signaling pathway, respectively.

### The hypothesis model of miRNAs medicated circadian rhythms and hippo signaling pathway

Taken together, there may be three models of the miRNAs to mediate the interaction between the circadian rhythms and hippo signaling pathway (Figure 5A). First model can be exemplified by miR-449a. CLOCK/ARNTL1 heterodimers can bind to the E-box in the upstream regulatory sequence and activate the expression of miR-449a, and miR-449a can act as a negative regulator of Per2 by targetting its 3′-UTR. The other targets of miR-449a, Ppp1ca may dephosphorylate casein kinase I ϵ (CKIϵ) Csnk1e to regulate the speed and rhythmicity of PER2 phosphorylation. In the second model, miRNAs mediate circadian rhythms and hippo signaling pathway through their complex target genes networks, like miR-125a-3p. MiR-125a-3p targets Per3 and Csnk1e, separately. And Csnk1e can regulate PER3 phosphorylation. In the third model, miRNAs are regulated by CLOCK/ARNTL1 heterodimers through E-box in their upstream sequence, and their target genes indirectly interact with circadian genes, such as miR-144, miR-199b*, and *miR-200a*.

**Figure 5:** Construct and validate the hypothesis model of miRNA-mediated circadian rhythms and hippo signaling pathway (**A**) The models of miRNA-mediated circadian rhythms and hippo signaling pathway. (**B**) Overexpression miR-449a down-regulate the expression level of PER2. (**C**) Inhibition miR-449a up-regulate the expression level of PER2. miRNAs compared with NC, antimiRNAs compared with anti-NC, *n*=3 of each group. *P<0.05.

### miR-449a regulates the expression level of PER2

To test the hypothesis model by overexpressing or inhibiting miRNA, we analyzed the regulatory effect of miR-199a-5p, miR-449a, and miR-96 on the expression of PER2 in NIH-3T3 cells. The expression level of PER2 was reduced by overexpression of miR-199a-5p and miR-449a (Figure 5B), and PER2 level was increased by inhibiting miR-449a with antagomirs (Figure 5C).

## Discussion

In the present study, we exploited the data from miRNAs microarray and identified the function of altered genes using bioinformatics analysis. To our knowledge, this is the first work to study *Clock* mutant effects on miRNAs expression in mouse SCN. Microarray analysis identified 39 significantly different expressed miRNAs, while miR-144, miR-199b*, miR-200a, miR-200b, miR-449a, and miR-96 were both changed at two different time points. Our results also showed that 12 of these miRNAs had the canonical E-box element. The pathways analysis suggested that the clock-regulated miRNAs at two different time points participated in many related or overlapping processes, even though they had only six miRNAs in common. Also the miRNAs influence extremely diverse processes.

The SCN has been reported to drive rhythms in behavior, physiology, metabolism, and hormone secretion via major output pathway, including autonomic neural connections and hormones, as well as less directly through circadian modulation of body temperature and feeding behavior [13,14]. The exception pathways related to metabolism and hormone secretion were evident, such as the biosynthesis, degradation, and metabolism of fatty acid, amino acid and steroid, and thyroid hormone signaling pathway. Also other canonical signaling pathways like Hippo, TNF, Foxo, Wnt, Hif-1, and AMPK signaling pathway were detected. Forkhead box class O3 (FOXO3) signaling was required for circadian rhythmicity in the liver via regulation of *Clock* [15]. The abilities of AMPK to mediate circadian regulation and of CRY1 to function as a chemical energy sensor suggested a close correlation between metabolic and circadian rhythms [16,17].

We focussed on the hippo signaling pathway, which regulate the animal organ development and growth. By further analysis, the gene *csnk1e*, also known as CKIϵ was a core gene to connect the circadian rhythms and hippo signaling pathway. In mouse, CKIϵ-binding domain and phosphorylation sites of PER proteins have been identified [18]. Moreover, CRY proteins protect PER from degradation, which form a CRY–PER–CKIϵ complex [19]. And this complex inhibits the transcriptional activity of the DNA bound BMAL1–CLOCK complex. Additionally, *CKIϵ* has been detected to be a target gene of miR-125a-3p in C2C12 cells by CLIP-seq [20]. miR-125a-3p–CKIϵ–PER–CRY–CLOCK complexes may be established in SCN and regulate SCN function. The τ mutation in the *CKIϵ* gene resulting in an exchange of the conserved amino acid residue 178 (R178C) have a shortened circadian period and CKIϵ plays an important role in neurodegenerative diseases [21]. Circadian biology is disrupted in a number of neurodegenerative diseases but the precise reasons for this remain unknown [22]. We suppose that the changing expression of miR-125a-3p–CKIϵ–PER–CRY–CLOCK complexes may be the reason of circadian disruption in neurodegenerative diseases. Recently, in the review of Lo Sardo and colleagues [23], they suggested a hypothesis that melatonin and hippo signaling pathway may have potential cross-talk. Melatonin is an indolic hormone that regulates circadian rhythms [24]. We predict that melatonin, miRNAs, CKIϵ, and core circadian genes may also have potential complex relation. Although these potential cross-talks need extensive experimental validation, they may open up a new field of investigation with important implications for better understanding circadian rhythms.

Interestingly, the results of pathway analysis showed that miR-125a-3p and miR-214 were implicated in every process. miR-125a-3p plays crucial roles in many different cellular processes like cell differentiation, proliferation, and apoptosis by targetting many different transcription factors, matrix-metalloprotease, growth factors, and so on [25]. miR-214 is deregulated in several human tumors including melanoma, breast, ovarian, gastric, and hepatocellular carcinomas [26]. And it contributed to the co-ordination of essential signaling pathways, such as the PTEN/AKT, β-catenin, or receptor tyrosine kinase pathways [27]. The fact that miR-125a-3p and miR-214 displayed in every process was most likely due to different mRNA targetting and/or target gene different expression in different processes. Although, there has been no report about the relations between miR-125a-3p/miR-241 and the circadian rhythms, we demonstrate that miR-125a-3p and miR-214 may play an important role in regulating the SCN function following *Clock* mutant.

The present results imply that a relatively large number of circadian expressing genes may possibly be regulated directly by *Clock* via the E box. The expression of miR-142-3p was under clock control. Further, chromatin immune precipitation (ChIP) assays showed that *Clock* was able to directly bind to the E-box in the upstream regulatory sequence of miR-142-3p [28]. The results of study the genes expression in liver of *Clock* mutant mice showed that both the *DBP* and *TEF* genes was depressed in *Clock* mutant mice, suggesting that the expression of these PAR basic leucine zipper transcription factors is positively regulated by CLOCK via E box elements *in vivo* [29]. The expression of miR-199a-5p, miR-200a, miR-200b, and miR-96 seems to be regulated indirectly by CLOCK in the mouse SCN. We concluded that clock-regulated miRNAs may have three models, suggesting a potential negative feedback loop consisting of the miRNAs and the circadian rhythms.

In conclusion, the present study demonstrates that *Clock* mutant causes modulation of miRNAs expression in the mice SCN. Bioinformatics function analysis demonstrates that clock-related miRNAs and their putative target genes may regulate the pathways that are important for SCN function. Taken together, the change in specific miRNAs levels in *Clock* mutant mouse indicates that the miRNAs, which serve as small players and have multiple functions, may be the key hub that connect circadian rhythms and other pathways via its complex target gene networks.

## Abbreviations

BMAL1: brain muscle arnt-like1
CKIϵ: casein kinase I ϵ
CLOCK: circadian locomotor output cycles kaput
qRT-PCR: quantitative real time polymerase chain reaction
MCODE: molecular complex detection
miRNAs: microRNAs
PPI: protein–protein interaction
SCN: suprachiasmatic nuclei
WT: wild-type
ZT: zeitgeber time
